The article "Effect of Thiopental on Ischemic Stroke in Rat Brain in Spontaneously Hypertensive Rats" was retracted in 2023. Reasons: signs of a paper mill; suspected computer-generated content; unreliable results or conclusions; concerns about the data.

# Effect of Thiopental on Ischemic Stroke in Rat Brain in Spontaneously Hypertensive Rats

**DOI:** 10.1155/2022/8063965

**Published:** 2022-01-22

**Authors:** Lu You, Qian Zhao, JianYong Yan, Wen Li, Ye Yang, Chenguang Qin

**Affiliations:** ^1^Department of Anesthesiology, Guizhou Provincial People's Hospital, China; ^2^Department of Anesthesiology, Guizhou Provincial Orthopaedic Hospital, China

## Abstract

*Motivation and Problem Statement*. Thiopental is an anesthetic drug related to the condition of controlling the area of neurological contexts. This study is related to the analysis of effectiveness for the condition of thiopental application on spontaneously hypertensive rats. *Methodology*. We have evaluated the thiopental induction as the anesthetic agent. The hypertensive rats were selected to administer thiopental in the form of anesthesia. The selection and application of hypertensive strokes are related to the derivation of an inducible model to assess the efficacy for analyzing the ischemic stroke parameters which relate to the human body. We used middle cerebral artery occlusion (MCAO) models related to spontaneous hypertension with the area of examining the complications in ischemic stroke. *Results and Conclusion*. The study focused on the experimental analysis based on the selection of spontaneously hypertensive rats associated with the incidence of ischemic stroke. Application of thiopental has reported the weak functionality and mechanism on the relaxation of neuronal activity in the case of rat brain. The considered population of the spontaneously hypertensive rats is evaluated based on the condition of effectiveness as well as the duration of the medication effects within the rat brain. Involvement of thiopental in the case of ischemic stroke has provided the area of risk development for high rate of death incidences after occurrence of acute ischemic stroke. A complication in the area of defining neuroprotective actions provides difficulty in drawing an appropriate conclusion of the study.

## 1. Introduction

Hypertension was not a treatable disease about half a century ago. However, today, it is a prevalent, noncommunicable chronic disease worldwide and could be inhibited by drugs [1]. Patients with hypertension had increased possibility of morbidity and mortality when undergoing anesthesia [2]. Thiopental is commonly known as thiopental sodium used as the anesthesia component, resulting in muscle relaxation. Moreover, it has been found that thiopental is used as an *adjunct* related to the anesthesia medicines to control the severe stroke complications. During the condition of ventilation and controlled interventions, thiopental sodium has been incorporated as maintaining the area of intracranial pressure increased among the patients of stroke [3]. Thiopental is related to the contraindications of respiratory obstruction as well as the condition of severe shock through the process of medicinal administration. Application of anesthesia in the case of relative context of the human stroke management and effects are yet to be highlighted through the research.

The article "Effect of Thiopental on Ischemic Stroke in Rat Brain in Spontaneously Hypertensive Rats" was retracted in 2023. Reasons: signs of a paper mill; suspected computer-generated content; unreliable results or conclusions; concerns about the data.

Thiopental as an anesthesia is related to the derivation of controlling the condition of the *systemic arterial blood pressure* including the context of *thermoregulation*. It has been reported that in the case of brain injury, anesthesia is directly involved with the prospects of controlling ischemic stroke, hemorrhagic stroke, pressure, and trauma [4]. Anesthesia associated with thiopental sodium has been considered as a difficult area of research to understand effectiveness on the ischemic stroke condition. The study is responsible for applying animal models through the involvement of hypertensive rats for thiopental application for controlling ischemic stroke.

## 2. Theory and Analysis

### 2.1. Unitary Theory of Anesthesia

A theory of the application in anesthesia is involved in the condition of controlling the process of relaxing nerves and muscles. According to the unitary theory of anesthesia, a physiological condition in the anesthesia is related to the understanding of specific issues related to the area of controlling the function of nerve cells. Application of the unitary theory has been responsible for defining the area of lipid membrane and their specific functions accumulated within the condition of thiopental sodium.

Based on the involvement of thiopental sodium as an anesthesia, a condition of the fluid-solid phase has been determined through the formulation of lipid membrane structural differentiation [5]. In the case of understanding the effectiveness of thiopental in anesthesia for ischemic stroke for the hypertensive, rats have defined the implementation of ion gate, binding of the transmitter, and transmitter influences on the synaptic region. Application of the unitary theory has defined that anesthesia resulted in the fluidization process of the nerve membranes along with the nervous system to provide the condition of resisting the phase separation of the membranes [6].

According to the development of the unitary theory, two different areas of the anesthesia application have been confined such as lipid theory and protein theory. Application of the lipid theory is responsible for defining the involvement of cell membrane controlling approach in the case of excessive pressure. Lipid theory defines that the anesthesia components such as thiopental dissolve within the lipid bilayer, responsible for formulating the management of the alternative physical properties within the nerve cell.

The article "Effect of Thiopental on Ischemic Stroke in Rat Brain in Spontaneously Hypertensive Rats" was retracted in 2023. Reasons: signs of a paper mill; suspected computer-generated content; unreliable results or conclusions; concerns about the data.

Changes in the physiological properties have been developed through the derivation of fluidity development followed by the volume increment within the cell membrane after dissolving the anesthetic components. Lipid theory has suggested the condition of the altered condition in the ion exchange activity associated within the cell membrane. Protein theory related to the anesthesia application and mechanism has reported the condition of volume expansion of the lipid membrane due to the dissolving process of the anesthetic substance. A process of transmission within the synapsis is developed through the correlation of the anesthetic components as well as the protein molecules. Thiopental as an anesthetic component is responsible for altering the application of the ion gating along with the channel of the protein receptors.

### 2.2. Theory of Neurophysiology Related to Anesthesia

According to the development of the theory of neurophysiologic condition in anesthesia, it is related to the area of determining suppressive awareness. Based on the administration of this theory, the neurophysiological area of anesthesia is related to the control and management of the depressive condition within the brain cells. In the case of hypertensive rats, application of thiopental as an anesthetic component acts on the *ascending reticular activating system* (*ARAS*) related to the portion of the cortex and thalamus of the rat brain [7]. Involvement of anesthesia within the brain cells of the hypertensive rats reflects the area of the neurophysiological space through the control and management of the pressurized conditions.

## 3. Method and Material

### 3.1. Design of Experiment

In this research, the condition of ischemic stroke has been considered to evaluate the process of thiopental induction as an anesthetic agent. In the design of the experiment, we have considered through the selection of the population or sample. In this research, we selected hypertensive rats for the area of the ischemic stroke related to the administration of thiopental in the form of anesthesia. According to the requirement of the research, potential hypertensive rats are examined through understanding the neurological complications in the rat brain after the condition of ischemic stroke [8].

The selection and application of the spontaneously hypertensive strokes are related to the derivation of an inducible model for assessing the effectiveness for studying the ischemic stroke parameters related to the human body. The experimental design for understanding the area of thiopental administration can be determined through the variation in the process of sacrificing the selected animals after growing the condition of stroke.

The article "Effect of Thiopental on Ischemic Stroke in Rat Brain in Spontaneously Hypertensive Rats" was retracted in 2023. Reasons: signs of a paper mill; suspected computer-generated content; unreliable results or conclusions; concerns about the data.

Neurological effectiveness of the rat brain has been considered through the implementation of thiopental on the area of ischemic stroke process. Moreover, spontaneous hypertensive rats are applied for the authentic stroke model to understand the area of anesthesia effectiveness on the brain cells of the rat. Middle cerebral artery occlusion (MCAO) models related to the spontaneous hypertensive rats are involved with the area of examining the complications in ischemic stroke [9].

### 3.2. Animal Model Description for the Study

In this study, an animal model has been applied for the derivation of the major context for analyzing effectiveness of thiopental associated with the condition in the ischemic stroke. *Spontaneously hypertensive rats* are considered for the animal model to understand the animal model based on the development of neurological deficits for the condition of developing ischemic stroke. Thiopental administration has been developed through the animal model to understand the functioning of the rat brain. Moreover, the pattern of the ischemic stroke is defined through the neurological complications related to the functioning in the rat brain.

Spontaneously hypertensive rats are considered through the animal model to define the condition of sacrificing state after developing the condition of ischemic stroke. The rat brain function based on the process of the anesthetic component such as thiopental was considered through the process of deriving middle cerebral artery (MCA) and relative condition of common carotid artery (CCA).

Administration of thiopental injection based on the anesthetic component was defined through the prospects of applying appropriate animal models to the area of research. The animal model based on the selection of ischemic stroke developing spontaneously hypertensive rats was derived through the area of defining the process of anesthetic activity.

### 3.3. Identification of Neurological Parameters

In this research, an animal model was selected for the area of considering the pattern of ischemic stroke report after administration of thiopental. Derivation of the neurological parameter as well as the symptoms is correlated to the condition of rat brain function associated with the ischemic stroke. Involvement of the process related to the muscle and nervous system relaxation procedure by thiopental related to the area of the ischemic stroke was defined through the neurological parameters.

Rat brain functioning has been determined through the induction of thiopental throughout the pattern of the neurological deficit model for the limb placement context. In the case of the spontaneously hypertensive rats developing ischemic stroke, two factors are determined such as motor functioning of the rat and somatosensory parameters related to the neurological complications.

The article "Effect of Thiopental on Ischemic Stroke in Rat Brain in Spontaneously Hypertensive Rats" was retracted in 2023. Reasons: signs of a paper mill; suspected computer-generated content; unreliable results or conclusions; concerns about the data.

### 3.4. Derivation of the Volume

It has been observed that the condition of the volume related to the nerve cell infarction has been considered for understanding the effectiveness for thiopental related to the ischemic stroke condition. Volume infarct derivation is related to one of the major components for understanding the area of muscle relaxation functions of the rat brain affected by ischemic stroke complications [10]. Infarct volume of the spontaneously hypertensive rat has been observed through the application of microscopy such as light microscopy. Changes in the volume have been defined through the involvement in the context of ischemic stroke factors.

### 3.5. Analysis

In this research, data analysis has been conducted through the implementation of the one-way ANOVA or analysis of variance. Data gathered from the experiment including changes in the infarct volume has been analyzed through the implementation of ANOVA [11]. Neurological parameters and relative complications have been derived through the identification and analysis of the variance. Infarct volume is the important factor related to the derivation in the effectiveness resulting from the application of thiopental as an anesthetic component for ischemic stroke.

## 4. Results

### 4.1. Effectiveness of Thiopental

Application of thiopental as an anesthetic agent has been associated with the process of developing unconsciousness among the patients. The considered population of the spontaneously hypertensive rats is evaluated based on the condition of effectiveness as well as the duration of the medication effects within the rat brain. Duration of the unconsciousness has been analyzed based on the implementation of thiopental as an anesthetic drug. It has been reported that thiopental has the potential to affect the body within 30 seconds. A single dose of the thiopental medicine has the capability to continue with the unconscious condition until 20 minutes to 30 minutes [3]. In the case of these spontaneously hypertensive rats related to the condition of ischemic stroke, thiopental rapid uptake has occurred in the vascular area of the rat brain.

In the case of spontaneously hypertensive rats selected for the research, thiopental sodium as an anesthetic drug has reported the area of the plasma protein and regulatory interactions to control the brain cells and tissues for relaxation (see Figure 1). Thiopental sodium has been observed as the major anesthetic drug related to the area of prolonged duration of the effectiveness. Time related to the unconsciousness mode involved with the area of thiopental sodium has resulted in a long activity of the anesthetic component in the case of spontaneously hypertensive rats with the condition of ischemic drug. The process of sacrificing the lives of the selected rats has reported that the death cases are related to the animals after injecting thiopental in the condition of ischemic stroke.

The article "Effect of Thiopental on Ischemic Stroke in Rat Brain in Spontaneously Hypertensive Rats" was retracted in 2023. Reasons: signs of a paper mill; suspected computer-generated content; unreliable results or conclusions; concerns about the data.

The nervous system of the thiopental-injected rats is determined through the relaxation in the signalling and synaptic transmitter for the prolonged duration of the unconsciousness related to the rats. Moreover, in the case of a few of the hypertensive rats, death cases occurred after the induction of thiopental after the condition of ischemic stroke. According to the result of death, events involved with the case of thiopental injection can provide the context of detrimental incidence regarding sodium thiopental incorporation. In the case of ischemic stroke related to the rat brain, effectiveness of thiopental is high in the condition of hypertensive rats.

### 4.2. Neurological Parameter

The selected spontaneously hypertensive rats are evaluated through the identification of neurological parameters to understand the thiopental mechanism and action in case of ischemic stroke related to the rat brain. Identification of the neurological parameter has been related to the condition analysis due to the induction of thiopental along with the context of limb placement in the case of hypertensive rats. Incidence of brain ischemia has been considered in the case of understanding neurological parameters related to the administration of thiopental related to the area of controlling ischemic stroke factors.

In this case, the best results related to the condition of neurological effectiveness have been developed through testing after 4 weeks of limb placement. Thiopental injection administration condition after 4 days of limb replacement provided the condition of poor neurological deficits related to the effects of the anesthetic components (Figure 2). Neurological activity within the hypertensive rat after 4 weeks of limb replacement provided the condition for weak functional activity after administration of thiopental. During the experiment, weak report of the thiopental performance has been reported for the context of limb replacement and neurological complications in the case of hypertensive rats.

### 4.3. Volume Analysis of Infarct

Size of the infarct analysis is related to the condition of defining mortality rate associated with the selected group of spontaneously hypertensive rats examined for ischemic stroke. In the case of ischemic stroke, infarct volume is related to the analysis of the condition for pathological test for the context of clinical deficits and complications. Development of the identification factor for the relative area of infarct volume has been identified through the administration of thiopental and effects for stroke management.

The article "Effect of Thiopental on Ischemic Stroke in Rat Brain in Spontaneously Hypertensive Rats" was retracted in 2023. Reasons: signs of a paper mill; suspected computer-generated content; unreliable results or conclusions; concerns about the data.

According to the involvement of thiopental injection, an enlarged volume of the infarct is located for the hypertensive rats related to the incidence of ischemic stroke. The results of enlarged volume in the infarct are related to the condition of defining relative loss of neuron from the rat brain after the administration of thiopental for ischemic stroke.

## 5. Discussion

The experimental report has suggested that thiopental is used in the case of anesthetic treatment, which resulted in a prolonged condition of unconsciousness among the hypertensive rats after ischemic stroke. According to the involvement of this specific drug component *sodium thiopental*, longer effectiveness of neurological and muscle relaxation has been reported for the area of ischemic stroke. Controversial analysis of the long-term effect of the thiopental drug on the condition of ischemic stroke has reported the area of weakness for the hypertensive rats. In this experiment, the situation of sacrificing the lives of selected animals reported that thiopental is related to the high incidence of death cases. Thiopental, as an anesthetic component, is related to the area of the selective mortality rate at a high scale after the condition of ischemic stroke. Rat brain analysis through the ischemic stroke is related to the condition of defining high risk of thiopental application [14].

Higher effectiveness of the thiopental medicine on the condition of ischemic stroke has resulted in the death cases associated with the area of controlling neurological functions. According to the involvement of thiopental as an anesthetic component among the rats, spontaneously hypertension has been reported in the area of lower rate of performance on rat brain [15]. Thiopental is an anesthetic drug component related to the area of a lower rate of recovery for the condition of postlimb placements in the case of ischemic stroke.

Application of anesthesia in the case of ischemic stroke management is related to the area of defining endovascular treatment and context of controlling the heart rates including pressure. Relaxing the neuronal activity is related to the evaluation of the anesthetics in postischemic stroke situations. Complexities have been present with the incorporation of thiopental related to the area of ischemic stroke resulting in the failure in acute circulatory functions [16]. Risks of ischemic stroke and the condition of cardiovascular disease have been involved with the high rate of mortality in the case of administering thiopental.

The article "Effect of Thiopental on Ischemic Stroke in Rat Brain in Spontaneously Hypertensive Rats" was retracted in 2023. Reasons: signs of a paper mill; suspected computer-generated content; unreliable results or conclusions; concerns about the data.

It has been observed that the patients dealing with acute ischemic stroke and condition of thiopental induction develop a risk of severe health outcomes. Induction of the general anesthesia related to the endovascular stroke condition has been reported in the area of anesthetic component application for controlling the neuroprotective functions of the drug components. Thiopental is related to the area of the lower rate of the neuroprotective functionality among the rat brain [17].

According to the application of the neuroprotective function by anesthesia, neurotransmitter suppression along with the *cerebral metabolic rate of oxygen* (*CMRO2*) reduction has been performed. Thiopental has been involved with the less potential for CMRO2 reduction and restriction of neurotransmitters to manage the area of ischemic stroke. A lower rate of the neuroprotective activity as a member of the *barbiturate* group has developed conflict for the controlling effect of neuronal functions.

A severe outcome along with the large volume of the infarct in the case of rat brain has been observed during the application of thiopental [18]. In the case, applying thiopental related to the area of longer time for the unconsciousness has been considered through the neuronal activity in thiopental.

A context of the longer period of hypertension among the selected animals has reported a higher risk potential related to the damaged condition of the brain cells [19]. The advantage is that thiopental is responsible for less effect on the context of damaging rat brain for lower rate of the involvement in focal cerebral ischemia for hypertensive rats. The limit is that a conflict has arisen with the implication of neuroprotective functionalities related to thiopental for acute ischemic stroke [20].

## 6. Conclusion

The study focused on the experimental analysis based on the selection of spontaneously hypertensive rats associated with the incidence of ischemic stroke and revealed that effectiveness of thiopental is high in the condition of hypertensive rats. More experiments are still needed to confirm this result.

## Figures and Tables

**Figure 1:** Sodium thiopental and effectiveness on the condition of the nervous system (source: [12]).

**Figure 2:** Sodium thiopental anesthetic effects related to the condition of arterial concentration and neurological activity (source: [13]).

The article "Effect of Thiopental on Ischemic Stroke in Rat Brain in Spontaneously Hypertensive Rats" was retracted in 2023. Reasons: signs of a paper mill; suspected computer-generated content; unreliable results or conclusions; concerns about the data.

## Data Availability

The data used to support this study is available from the corresponding author upon request.
